# A New Strategy Using ALDH^high^-CD8+T Cells to Inhibit Tumorigenesis

**DOI:** 10.1371/journal.pone.0103193

**Published:** 2014-08-08

**Authors:** Huiyan Luo, Changqing Zeng, Cheng Fang, Sharvesh Raj Seeruttun, Lin Lv, Wei Wang

**Affiliations:** 1 Department of Oncology, the Third People's Hospital of Chongqing, Chongqing, P. R. China; 2 Department of Gastrointestinal Surgery, Fujian Provincial Hospital, Fuzhou, P. R. China; 3 Provincial Clinical Medical College of Fujian Medical University, Fuzhou, P. R. China; 4 Department of Gastric and Pancreatic Surgery, Sun Yat-sen University Cancer Center, Guangzhou, P. R. China; 5 State Key Laboratory of Oncology in South China, Guangzhou, P. R. China; 6 Collaborative Innovation Center for Cancer Medicine, Guangzhou, P. R. China; 7 Department of Medical Oncology, Guangzhou First People's Hospital, Guangzhou, P. R. China; University of Birmingham, United Kingdom

## Abstract

**Background:**

Currently, many studies suggest that cancer stem cells (CSCs) are responsible for tumor initiation, tumorigenesis, metastasis and recurrence. CSCs have been identified from various human and murine tumors. The identification of CSCs allows us to develop strategies to target the CSCs.

**Methods and Results:**

In this study, we used ALDEFLUOR as a single marker to isolate the CSCs from the human lung cancer cell line H460. We then characterized the CSCs by testing their sphere formation ability and tumorigenicity. Furthermore, we used CSC lysate-pulsed dendritic cells to stimulate CD8+T cells as a treatment strategy. Our study demonstrated that ALDEFLUOR could be used as a single marker to identify CSCs from the human lung cancer cell line H460. The ALDH^high^ cells could form more spheres and were more tumorigenic than the ALDH^low^ cells. Further study demonstrated that ALDH^high^-CD8+T cells conferred more significant antitumor effects, resulting in the inhibition of tumor growth and prolonged survival. And the ALDH^high^-CD8+T cells-mediated anti-tumor immunity might be due to the directly targeting against ALDH^high^ cancer stem cells (CSCs).

**Conclusions:**

This study shows that ALDH^high^-CD8+T cells mediate anti-tumor immunity by selectively targeting cancer stem cells, which result in inhibiting tumor growth and prolonging the survival of tumor-bearing mice, which provides a new strategy using ALDH^high^-CD8+T cells to treat tumors.

## Introduction

Lung cancer is considered the leading cause of cancer-related death worldwide. More than one million cases of lung cancer are diagnosed each year. Non-small cell lung cancer (NSCL) is the major type of lung cancer and accounts for approximately 80–85% of all lung cancers [1], [2]. Despite the development of surgery, chemotherapy and radiotherapy, the outcomes of lung cancer patients are still unsatisfactory. Even epidermal growth factor receptor (EGFR) tyrosine kinase inhibitors are only effective in a small population of lung cancer patients [3]. Many patients still develop distant metastasis and relapse after the traditional and target therapy [3]–[5]. Therefore, it is of great importance to know more about the lung cancer and to explore more effective therapeutic targets.

Tumor immunotherapy, which is the fourth strategy to treat cancer patients, has been developed in recent decades and has been reported to be an effective and promising method to treat cancer patients [6], [7]. The administration of dendritic cells and T lymphocytes has been used to treat certain cancers, such as melanoma, breast cancer and squamous cell carcinoma. However, only a small percentage of patients benefit from these immune therapies [8]–[10]. The treatment failure may be because these immune strategies are designed to target differentiated antigens. However, due to the heterogeneity of the tumor mass, the tumor cells have different differentiation and proliferation capabilities, which can lead to different prognoses [11]. The presence of cancer stem cells in the tumor residue largely contributes to tumor heterogeneity [12]–[14]. CSCs express undifferentiated antigens, and thus, these cells escape the interventions of the current immunotherapies.

Although there is only a very small percentage of cancer stem cells in the tumor mass, the CSCs are responsible for tumorigenesis, metastasis and relapse [15]. These cells are characterized by their ability to self-renew, their chemo- and radio-resistance, and their enhanced tumorigenicity [11], [16]–[18]. Thus, methods designed to target cancer stem cells may be more beneficial.

ALDEFLUOR/ALDH has been used as a single marker to isolate cancer stem cells from both human and murine tumors [3], [15], [19]–[22]. Some studies have reported that the ALDH-enriched cell population could be used as a source of antigens for the development of immune strategies to mediate tumor regression [23], [24]. Ning et al. used an ALDH^high^ CSC-pulsed dendritic cell vaccine to prevent tumor development and the lung metastases of squamous cell carcinoma and melanoma [23]. Visus et al. reported that adoptive transferred ALDH1A1-specific CD8+T cells could target the ALDH^bright^ cells, inhibit subcutaneous tumor growth, prevent metastasis and prolong the survival of the tumor-bearing mice [24].

Thus, in this study, we used ALDH as a single marker to identify and isolate cancer stem cells from the human lung cancer cell line H460. The characteristics of this ALDH^high^-enriched CSC population were verified by studying their sphere formation ability and tumorigenicity. We then used CSC lysate-pulsed dendritic cells as the antigen-presenting cells to stimulate purified CD8+ T cells. Tumor-bearing nude mice were treated with the different antigen-pulsed dendritic cell-primed CD8+T cells, and we assessed the therapeutic efficacy of the adoptive transfer of CD8+T cells by monitoring the s.c.tumor volumes and the overall survival.

## Materials and Methods

### Ethics Statement

All the mice were housed in specific pathogen-free condition at the Sun Yat-Sen University Cancer Center Animal facilities. The mice used for experiments were at the age of 7∼8 weeks. Mice exhibiting rapid weight loss, rough hair coat, hunched position, labored breathing, lethargy, difficulty with ambulation, ulcerated tumors that were bleeding, infected, or necrotic were humanely euthanized using CO2. All animal experiments were approved by the Institutional Review Board of the Ethics Committee of Sun Yat-Sen University Cancer Center.

### Cell line and culture

The human lung cancer cell line H460 was obtained from the American Type Culture Collection (ATCC) and cultured in RMPI-1640 medium supplemented with 10% heat-inactivated fetal bovine serum (FBS), 100 g/mL streptomycin, 100 U/mL penicillin, and 0.5 g/mL fungizone.

### Mice

BALB/c nu/nu mice were purchased from the Chinese Academy of Military Medical Sciences (Beijing, China); the mice used in these experiments were between 6 and 8 weeks of age.

### Preparation of primary tumor cells

The BALB/c nu/nu mice were challenged with 1×10^6^ H460 cells in the right flanks. On day 20, the freshly s.c tumors were collected and digested into single cell suspension using the enzyme digestion solution. Then the freshly harvested primary tumor cells were used for the detection of ALDH activity.

### ALDEFLUOR assay

The ALDEFLUOR kit (Stem Cell Technologies, Vancouver, Canada) was used to identify and isolate cancer stem cells from the human lung cancer cell line H460 and freshly harvested primary tumor cells according to the manufacturer's instructions. Briefly, the sample cells (1×10^6^cell/ml) were stained with ALDEFLUOR. Cells treated with the ALDH inhibitor diethylaminobenzaldehyde (DEAB) and stained with ALDEFLUOR were used as a negative control, and 7-ADD was used to assess cell viability. The identification and sorting of the CSCs were performed using a FACStarPLUS.

### Sphere culture

A total of 10,000 isolated ALDH^high^ CSCs were plated in ultra-low attachment plates and cultured in serum-free culture medium, which consisted of MEBM supplemented with 10 g/ml EGF, 1 mg/ml insulin, B27, and 1 mg/ml hydrocortisone. The ALDH^low^ non-CSCs were used as the control. The numbers of the spheres were calculated under the microscopy. The experiments were repeated at least 3 times, and each sample was set triplicated.

### Tumorigenicity of the ALDH^high^ CSCs

An equal number of isolated ALDH^high^ and ALDH^low^ cells (50,000 cells in 100 µl PBS) were mixed with Matrigel (1∶1, BD Biosciences, Bedford, MA). The mixed cells were then injected into the opposite sides of the flanks of the nude mice. The tumor sizes were monitored 3 times per week. Each group contains 3∼5 mice. And the experiments were repeated at least 3 times.

### Tumor cell lysate preparation

To prepare the tumor cell lysate used to pulse the dendritic cells, unsorted H460 cells, isolated ALDH^high^ or ALDH^low^H460 cells were resuspended at a concentration of 1 million cells in 1 ml of culture medium. After five rapid freeze-thaw cycles in a 37°C water bath and liquid nitrogen, the tumor cell lysates were stored at −80°C for later use.

### Cancer stem cell lysate-specific CD8+ T cell preparation

Peripheral blood mononuclear cells (PBMCs) were isolated from the peripheral blood of healthy donors using Ficoll-density gradient centrifugation as previously described [25]a. The mononuclear cells were plated in culture flasks in Quantum 007 medium (PAA, Pasching, Austria) at 37°C for 20 min. The non-adherent cells were collected and purified using CD8+ microbeads (Life Technologies, Shanghai, China) according to the manufacturer's instructions. Then, the purified CD8+ T cells were cultured in Quantum 007 medium containing 20 U/ml IL-2, 100 U/ml penicillin and 100 mg/ml streptomycin and were used for subsequent experiments. The adherent cells were cultured in RMPI-1640 supplemented with 10% FBS, 1,500 U/ml granulocyte macrophage colony-stimulating factor (GM-CSF; Peprotech, Suzhou, China), 500 U/ml interleukin-4 (IL-4; Life Technologies), 100 U/ml penicillin and 100 mg/ml streptomycin. The culture medium was half changed on day 3. On day 5, the non-adherent and loosely adherent DCs were harvested and counted. The DCs were then plated in 6-well plates with unsorted, ALDH^high^ or ALDH^low^H460 cell lysates at a 3∶1 ratio. After incubation for 24 hours, the unsorted tumor cell lysate-pulsed DCs, the ALDH^high^ tumor cell lysate-pulsed DCs and the ALDH^low^ tumor cell lysate-pulsed DCs were co-cultured with CD8+ T cells for 7 days to generate H-CD8+T, ALDH^high^-CD8+T, and ALDH^low^-CD8+T cells, respectively.

### Treatment protocol

The unsorted H460 cells were injected into the right flank of nude mice on day 0. Then, the mice were intravenously treated using various generated CD8+T cells 24 hours after the s.c.tumor challenge. The CD8+T cell administration was repeated twice, which were on days 8 and 15. Each mouse was treated with 1 million CD8+ T, ALDH^high^-CD8+ T or ALDH^low^-CD8+ T cells. The tumor sizes were measured 3 times per week. The overall survival was recorded until the mice met the endpoint requirements. Each group contained 3∼5 mice. And the experiment was repeated 3 times.

### Cytotoxicity assay

The cytotoxicity of the effect T cells against ALDH^high^ H460 cancer stem cells or H460 tumor cells were tested using the LDH-release assay (CytoTox 96 Non-Radioactive Cytotoxicity Assay, Promega, Madison, WI) according to the manufacturer's protocol. Briefly, the sorted ALDH^high^ H460 cells or unsorted H460 cells were seeded in 96-well round bottom cell culture plates at a density of 1×10^4^ cells/50 µl in a complete culture medium. Then the H-T, ALDH^high^-T or ALDH^low^-T were seeded at ratios of effect to target = 30∶1, 10∶1 and 3∶1. After 12 h of incubation, the cytotoxicity was assessed using Lactate Dehydrogenase (LDH) activity. The experiments were repeated at least 3 times by using effect T cells generated from various individuals.

### Statistical analysis

The data were analyzed using GraphPad Prism 5 (GraphPad software). The significance of the differences in tumor size, sphere formation, tumorigenicity and cancer stem cell lysis by effect T cells were evaluated using an unpaired Student's t-test. Survival analysis was determined using the log-rank test. A two-tailed *P* value <0.05 was considered significant.

## Results

### Isolation and identification of cancer stem cells using ALDEFLUOR as a marker

ALDEFLUOR/ALDH has been generally used as a single marker to identify cancer stem cells from both human and murine tumors, such as melanoma and breast cancers [20], [23]. By performing this technique, an enriched CSC population was isolated from the human lung cancer cell line H460. As shown in Figure 1A, approximately 10% of the tumor cells were ALDH^high^. The remaining 90% of the cells belonged to the ALDH^low^ population. Using a flow cytometry sorting technique, we isolated an equal percentage of ALDH^high^ cells and ALDH^low^ cells to further verify the cancer stem cell characteristics of the enriched ALDH^high^ population. Similarly, the presence of the ALDH^high^ subpopulation cells in established murine tumors was confirmed by analyzing freshly harvested tumor cells from *in vivo* established H460 murine tumors. After being digested into single cell suspensions, the ALDEFLUOR assay and flow cytometry were performed to verify the activity of ALDH in the xenograft. As shown in Figure 1B, around 6% of the freshly harvested tumor cells were the ALDH^high^ subpopulation.

**Figure 1:** The identification of ALDH^high^ cells from the human non-small cell lung cancer cells and primary tumor cells. ALDEFLUOR was used as a single marker to identify the ALDH^high^ cells from the H460 cell line (A) and freshly harvested tumor cells (B). Tumor cells incubated with both ALDH and DEAB were used as a negative control.

### Sphere formation of the ALDH^high^-enriched population

CSCs are characterized by their sphere formation ability, tumorigenesis and self-renewal. To verify whether the ALDEFLUOR-enriched population contained cancer stem cell-like cells, we first performed the sphere formation assay by culturing the ALDH^high^ cells in serum-free medium; the ALDH^low^ cells were also cultured under these conditions and were used as a negative control. Compared to the ALDH^low^ cells, the ALDH^high^ cells had an enhanced sphere forming ability. Figure 2A and B show representative pictures from the ALDH^high^ and ALDH^low^ cells on day 14. We also counted the numbers of the spheres formed by ALDH^high^ or ALDH^low^ H460 cells. As shown in Figure 2C, compared to ALDH^low^ H460 cells, the enriched ALDH^high^ H460 cells could form much more spheres (Figure 2C, *P* = 0.0034).

**Figure 2:** Sphere formation of the ALDH^high^ and ALDH^low^ cells. A total of 10,000 isolated ALDH^high^ or ALDH^low^ cells were cultured in serum-free medium. The representative photographs from the ALDH^high^ cells (A) and ALDH^low^ cells (B) were taken on day 14. The ALDH^high^ cells could form much more spheres than the ALDH^low^ H460 cells (C). The number of spheres were expressed as Mean± SEM, n = 4.

### Tumorigenicity of the ALDH^high^ cells in nude mice

It has been reported that cancer stem cells are more capable of forming tumors than unsorted tumor cells. A very small number of CSCs can form tumors. To test this hypothesis, an equal number of ALDH^high^ cells and ALDH^low^ cells were subcutaneously injected into the opposite flanks of nude mice. After the tumor cells were injected, both the ALDH^high^ and ALDH^low^ cells developed into a tumor mass. However, the volumes of the tumors generated from the ALDH^high^ cells were much larger than the tumors generated from the ALDH^low^ cells (Figure 3A, *P* = 0.0003)). Figure 3B–D show the representative growth curves of the tumors from 3 different mice. These data suggest that the ALDH^high^H460 tumor cells were much more tumorigenic than the ALDH^low^ cells.

**Figure 3:** Tumorigenicity of the ALDH^high^ and ALDH^low^ H460 cells. An equal number of ALDH^high^ and ALDH^low^ cells were inoculated into the opposite flanks of the same individuals. The sizes of the tumors were measured 3 times per week. (A) The tumor sizes of mice subjected to ALDH^high^ H460 cells were much more larger than the ALDH^low^ H460 cells. (B–C) show the representative tumor growth curves from 3 different mice.

### CSC-based CD8+ T cells confer significant anti-tumor immunity

Compared to the traditional whole tumor cell lysate-pulsed dendritic cell vaccine, the CSC lysate-pulsed dendritic cell vaccine exerts a more effective anti-tumor immunity [23]. Thus, in our research, we used the ALDH^high^ H460 CSCs as an antigen source to pulse the dendritic cells and generate CSC-based dendritic cells. Then, the CSC-based DCs were co-cultured with purified CD8+ T cells for 7 days. Here, we refer to the CD8+ T cells stimulated with the ALDH^high^ lysate-pulsed DCs as ALDH^high^-CD8+T. The CD8+ T cells stimulated by dendritic cells pulsed with the heterogeneous unsorted tumor cell lysate (H-CD8+ T) or the ALDH^low^ tumor cell lysate (ALDH^low^-CD8+ T)) were used as controls.

The treatment scheme is shown in Figure 4A. Unsorted H460 cells (1×10^5^) were subcutaneously injected into mice on day 0. The tumor-bearing mice were intravenously immunized with ALDH^high^-CD8+T, H-CD8+T, ALDH^low^-CD8+T or PBS (i.v.) three times at 1 week intervals(days 1,8 and 15).

**Figure 4:** ALDH^high^-CD8+ T treatment inhibits subcutaneous tumor growth. (A) The treatment scheme. (B) The tumor sizes of the mice treated with ALDH^high^-CD8+ T cells were much smaller than the tumors of mice treated with PBS, H-CD8+ T, or ALDH^low^-CD8+ T cells.

The tumor sizes were monitored until the mice met the endpoints. While the H-CD8+T or ALDH^low^-CD8+T could not significantly inhibit tumor growth, administration of the ALDH^high^-CD8+T cells could significantly inhibit tumor growth (*P*<0.05, compared to all other groups, Figure 4B).

The mice that were euthanized or died were both counted to assess the survival rate. As shown in Figure 5, the mice subjected to the ALDH^high^-CD8+ T cells had a longer survival time than mice subjected to PBS, H-CD8+T or ALDH^low^-CD8+Tcells (*p*<0.01, *p* = 0.01, *p* = 0.01, respectively, Figure 5). Additionally, the H-CD8+T or ALDH^low^-CD8+T treatments only had a 2–3 day advantage in the overall survival compared to the PBS treatment. The ALDH^high^-CD8+T treatment had a 13 day advantage over the PBS treatment in the overall survival (Figure 5).

**Figure 5:** ALDH^high^-CD8+ T treatment prolongs the overall survival of the tumor-bearing mice. The mice treated with ALDH^high^-CD8+ T cells survived much longer than the mice treated with PBS, H-CD8+ T, or ALDH^low^-CD8+ T cells.

To study the underlying mechanism of the anti-tumor immunity of the ALDH^high^-CD8+ T cells, we studied the cytotoxicities of the effect T cells in vitro. These activated effect T cells were assessed for cytotoxicity against ALDH^high^ H460 cells or unsorted H460 tumor cells. ALDH^high^-CD8+ T killed H460 CSCs efficiently and significantly more than H- CD8+ T (Figure 6A, *P* = 0.0011) and ALDH^low^- CD8+ T (Figure 6A, *P*<0.0001). Concurrently, the killing of unsorted H460 cells by ALDH^high^-CD8+ T was significantly less effective compared with both H- CD8+ T and ALDH^low^- CD8+ T (Figure 6B, *P*<0.0001). As shown in Figure 6C, the ALDH^high^-CD8+ T could kill much more ALDH^high^ H460 cells than unsorted H460 tumor cells (*P*<0.0001). These date suggested that the enhanced ALDH^high^-CD8+ T-induced anti-tumor immunity might be due to directly and selectively targeting of CSCs.

**Figure 6:** Cytotoxicities of effect T cells against cancer stem cells and tumor cells. The killing was measured by an LDH release assay as described in the Materials and Methods. Higher % of cytotoxicity means more cell lysis. (**A**) Cytotoxicities of CSCs mediated by the H-T, ALDH^low^-T and ALDH^high^-T are shown. (**B**) Cytotoxicities of unsorted H460 cells mediated by the H-T, ALDH^low^-T and ALDH^high^-T are shown. (C) ALDH^high^-T could kill much more CSCs than unsorted tumor cells.

## Discussion

It is generally accepted that the existence of cancer stem cells in the tumor mass are responsible for carcinogenesis, tumor maintenance, metastasis and relapse. Tumor relapse after surgery is largely due to the existence of these cancer stem cells in the residual tumor tissue or the circulating system [12]–[15]. Additionally, these cells are thought to be resistant to chemotherapy and radiotherapy [16], [17]. Most of the current immune strategies are designed to target differentiated antigens. However, cancer stem cells may not express these differentiated antigens and therefore may not be targeted by these strategies.

ALDEFLUOR has been used as a single marker to identify cancer stem cells from both human and murine cancers. Some studies have identified cancer stem cells from both human and murine lung cancers using ALDH as a single marker [3], [5]. However, these studies did not verify the stem cell characteristics of the ALDH^high^-enriched population. In this study, we used ALDH as a single marker to identify cancer stem cells from the human non-small cell carcinoma cell line H460 and freshly harvested primary tumor cells. Approximately 10% of the H460 tumor cells highly expressed ALDH. About 6% of the freshly harvested tumor cells are ALDH^high^ subpopulation. Both the ALDH^high^ and ALDH^low^ cells were isolated to verify their sphere formation abilities and their tumorigenicity. By culturing the isolated cells in serum-free culture medium, we found that the ALDH^high^ H460 cells could form more spheres than the ALDH^low^ cells. Another important characteristic of cancer stem cells is their strong tumorigenicity. After being challenged with an equal number of ALDH^high^ and ALDH^low^ cells in the same individuals, the ALDH^high^ cells developed larger tumors than the ALDH^low^ cells. The results from the sphere formation and tumorigenicity assays suggested that, compared to the ALDH^low^ cells, the ALDH^high^-enriched cells possessed more cancer stem cell abilities.

It is generally thought that the presence of CSCs in the bulk tumor mass may adversely affect the therapeutic efficacy of immunotherapies, thus leading to tumor recurrence, distant metastasis and treatment failure in most patients. Thus, the inability of traditional immune strategies to selectively target CSCs encouraged us to develop a more effective strategy that could specifically target CSCs, which may be an effective way to prevent tumor recurrence and metastasis.

Some studies using CSC-associated antigens to generate effect or T cells or to prime DCs have used antigens that have been verified as playing significant roles in tumor protection. Adoptive therapy with ALDHA1 peptide specific CD8^+^T cells resulted in the inhibition of tumor growth and metastasis, as well as a prolonged survival rate of the xenograft-bearing immunodeficient mice, according to Visus et al. [24]. Garcia-Hernandez et al. demonstrated that a prostate stem cell antigen (PSA)-based vaccine resulted in long-term protection against prostate cancer development, with a 90% survival rate at 12 months of age [26]. Duarte et al. used a CSC-enriched lysate from the rat PROb colon carcinoma cell line as a vaccine, and this CSC lysate derived-vaccine prevented the development of half of the liver metastases and resulted in a 99.5% reduction in tumor volume compared to the PBS-treated group [27]. Their studies suggest that cancer stem cell based immunotherapies show promising effect in cancer treatment.

In the current study, we used different antigen-pulsed dendritic cells to stimulate CD8+ T cells. Compared to PBS, H-CD8+ T and ALDH^low^-T, treatment with the ALDH^high^-T cells resulted in more significant anti-tumor immunity, which was evident by its inhibition of subcutaneous tumor growth and the prolonged overall survival. Further in vitro studies demonstrated that ALDH^high^ cancer stem cells could be efficiently and significantly destroyed by ALDH^high^-T cells. And the ALDH^high^-T cells could kill much more ALDH^high^ cells than unsorted H460 cells. These data suggested that the anti-tumor immunity of ALDH^high^-T might be due to the selectively and directly targeting CSCs. The immunological targeting of CSCs may provide a novel strategy for the development of more effective cancer immunotherapies.

Our current study found that ALDH^high^-T conferred more effective tumor protection, and these results provided more support for the use of ALDH^high^-T cells in combination with other therapies in treating established tumors, such as the administration of ALDH^high^-T cells after surgical excision of a s.c. tumor, as well as the combination of ALDH^high^-T cells with chemotherapy or radiotherapy.
